# The Effect and Mechanism of Exercise Training on Rats with Poststroke Depression Based on the Intestinal Flora

**DOI:** 10.1155/2021/3567447

**Published:** 2021-12-24

**Authors:** Jiaen Yang, Guangjin Zhou, Zixuan Ou, Ning Jia, Dong Wang

**Affiliations:** ^1^Department of TCM Rehabilitation Medicine, Affiliated Foshan Gaoming Hospital of Guangdong Medical University, Foshan, 528000 Guangdong, China; ^2^Department of Rehabilitation Medicine, Affiliated Hospital of Chengdu University, Chengdu, 610000 Sichuan, China

## Abstract

Depression of poststroke depression (PSD) is the most common neuropsychiatric complication after stroke. Patients with PSD had higher mortality, more cognitive disorder, lower quality of life, and higher suicidal tendency. The pathogenesis of PSD mainly involves neurotransmitter inflammatory factors, HPA and BDNF. Enteral dysfunction and intestinal flora disorders caused by stroke can participate in the pathogenesis of PSD through various ways, such as immune, endocrine, and nervous system. In this experiment, we used exercise training as an intervention means to explore the curative effect and possible mechanism by observing the changes of behavior, inflammatory factors, and intestinal flora in rats. The results show that the mechanism of exercise training to improve the depressive behavior of rats may be related to inhibiting the expression of proinflammatory factors and increasing the number of lactic acid bacteria in the intestine.

## 1. Introduction

The intestinal flora has a great impact on human health; it is involved in the central nervous system movement and has a certain impact on depression after stroke. The intestinal flora provides an important way to maintain body's immunity and delay the metabolism in the body. This article has practical significance for the research on the treatment of sports training in poststroke depression.

Based on the intestinal flora, there are many theoretical results in the study of the effect and mechanism of exercise training on rats with poststroke depression. For example, Huang Xiaoqun stated that the presence of the gut-brain microbiota axis enables the gut microbiota to effectively participate in the regulation of complex physiological processes in the body, and the precise coordination of the neuroimmune endocrine system enables the continuous participation of the gut microbiota. Regulate the central nervous system in the process [1]. Liu et al. studied the mechanism of compound Yinao Jieyu treatment of stroke stress rats from the perspective of changes in intestinal flora [2]. Miao and Lv observed the effect of Xingnaojing injection on the behavior of rats in the poststroke depression model and explored the related pharmacological mechanisms [3]. This article also conducted related research to explore the mechanism of intestinal flora in the treatment of PSD in sports training.

## 2. Based on the Intestinal Flora to Explore the Effect and Mechanism of Exercise Training on Rats with Poststroke Depression

### 2.1. Intestinal Flora

#### 2.1.1. Gut Microbes

Humans and microbial communities have formed a symbiotic relationship for a long time and a large number of microbes parasitize the skin, oral cavity, reproductive system, intestinal tract, etc. [4, 5]. It plays a very important role in the physiology, reproduction, immunity, metabolism, and evolution of the human body. Intestinal flora is the general term for all microorganisms coexisting with humans in the human gastrointestinal tract. The intestinal flora has many types and huge numbers, and its total weight is approximately similar to that of the liver, and its structure is also very complex.

Hundreds of millions of bacteria live in the human intestine. The ecosystem formed by these bacteria affects many physiological functions of the host, including important effects on brain function and development. It has always been thought that the intestine and the brain interact through the brain-gut axis, and this interaction may be caused by different types of nerves, endocrine systems, and immunity [6, 7].

The intestinal flora is divided into three categories: the first category, commonly known as “probiotics,” is a well-known functional flora that parasites in the human gastrointestinal tract and is beneficial to the human body. These flora can help the human body to synthesize vitamins and promote the absorption of protein and inorganic substances. The second category is commonly known as “harmful bacteria.” As the name suggests, these bacteria can hinder the normal physiological functions of the human body, produce harmful substances, and even cause physical diseases. The third type of bacteria is neutral bacteria. Neutral bacteria do not cause harm or benefit to the human body. Most of them do not parasitize in the intestine for a long time, and they account for a very small proportion of the intestinal flora. Once the human intestinal environment changes or the immunity declines, the normal physiological balance of the intestinal environment is broken, and the ratio of harmful bacteria to neutral bacteria will increase, resulting in imbalance of the intestinal flora. At this time, the harmful substances produced by the metabolism of pathogenic bacteria and neutral bacteria increase, which may make people sick.

It was found that Enterobacteriaceae and Veroniaceae increased in the high incidence of stroke, and the content of Triconaceae and Wuctinaceae that produce SCFAs decreased [8]. Exercise deficiency, intestinal flora disorders induced by stress events, and intestinal inflammation can cause dyslipidemia and participate in the occurrence and development of hypertension and diabetes [9, 10]. In addition, the intestinal flora can promote atherosclerosis formation and development through inflammation, lipid metabolism, and trimethylamine-N-oxide (TMAO) production [11].

After stroke, the inflammatory response can destroy the homeostasis of the intestinal barrier and intestinal flora, and the endotoxins and inflammatory factors entering the blood through the intestinal barrier can damage the blood-brain barrier and aggravate the oxidative stress of the brain tissue [12, 13]. Activated HPA axis and sympathetic nerves can exacerbate intestinal dysfunction, inhibit the synthesis of intestinal neurotransmitters and nerve conduction, lead to poor prognosis of stroke, and increase the risk of psychiatric diseases after stroke. Studies have found that Lactobacillus not only can improve vascular endothelial function and reduce the risk of stroke but also can inhibit oxidative stress and nerve cell apoptosis and reduce the degree of stroke damage [14, 15].

### 2.2. Poststroke Depression

Stroke is one of the diseases threatening human health, and the incidence has been on the rise in recent years. At present, the incidence of the disease is increasing year by year with the aging of the population, and there is a trend of younger development. Poststroke depression (PSD) is a relatively common cerebrovascular event; it mainly occurs after a stroke [16, 17] and also can cause depression, depression, listlessness, and even insomnia. Depression is very likely to occur in the acute and recovery phases of stroke. Depression is the result of damage to various areas of the brain involved in emotional control or long-term negative external stimulation, which leads to changes in neuronal degeneration and neuroplasticity in this area, especially the hippocampus of the brain [18].

One of the main complications of stroke is poststroke depression. PSD can not only significantly affect the quality of life, leading to various negative emotional experiences, but also the recovery of neurological function, thus increasing the length of hospitalization, disability rate, mortality, and relapse rate, with serious negative effects on patient's disease. [19] Compared with primary depression and other secondary depressions, there are certain differences in the etiology, pathogenesis, clinical manifestations, course and prognosis, diagnosis, and treatment of poststroke depression. However, the characteristics of depression are different among PSD populations of different ages, genders, and PSD individuals. The disease that occurs has a serious impact on the quality of life of stroke patients and also brings various adverse effects to the families of such patients, and delays in patients with neurological deficits are not conducive to their normal ability recovery, resulting in various negative consequences.

1. The pathogenesis factors and pathogenesis of PSD are very complex. At present, there is no unified understanding of the pathogenesis of PSD, which mainly includes response mechanisms, internal spontaneous mechanisms, and comprehensive biological-psychological-social feedback mechanisms. The clinical symptoms of PSD are rich and diverse, and it is difficult for one scale to fully assess all clinical symptoms groups; therefore, in clinical studies of PSD, different tools and scales are often used to evaluate patients, or multiple scales simultaneously. These scales were evaluated, and given the different evaluation contents and methods, the evaluation results may also differ when different evaluation tools are used, and individuals with different clinical characteristics also need to develop different treatment options. Poststroke depression is an important psychological sequelae of ischemic stroke. About one-third of different stroke patients are affected by it. Poststroke depression can increase the morbidity and mortality of patients. Therefore, it is of very important significance to develop effective identification and treatment of poststroke depression
2. The main manifestations of early poststroke depression are depression, restlessness, and autonomic symptoms. The risk of poststroke depression runs through the early, middle, and late stages of stroke. Poststroke depression is related to the level of physical impairment, cognitive impairment, and stroke severity
3. Treatment methods for poststroke depression

Some treatments have been proven to be potential treatments for poststroke depression.

1. Antidepressant treatment can improve brain executive ability after stroke. One is through the cortex-striatum-globus pallidus-thalamus-cortex pathway, and the other is through the reorganization of brain-derived neurotrophic factors and reorganization of neural pathways. Another mechanism by which antidepressants work is nerve regeneration
2. Psychotherapy interventions include cognitive behavioral therapy, social work interventions, service suggestions, and consultations. Psychotherapy is effective in the prevention and treatment of poststroke depression and has been recognized as a preferred treatment option in the community and other clinical patients (such as myocardial infarction)
3. Electroconvulsive therapy is often used to treat patients with persistent major depression and electrically induced epilepsy. Electroconvulsive therapy is an effective treatment for depression
4. The music therapy group is more conducive to the recovery of cognitive functions including oral memory and concentration and can improve mood
5. High-intensity exercise training can increase the level of brain-derived neurotrophic factors in normal adults

### 2.3. Sports Training

Long-term and adequate exercise training can improve learning and memory ability and have a positive effect on depression. Brain-derived neurotrophic factor is a protein with the activity of promoting nerve growth and has an important effect on neuron development, survival, growth, differentiation, and plasticity of neurons. Regular and sufficient exercise training can increase the brain-derived neurotrophic factor of hippocampus, thereby improving the condition of poststroke depression. However, the method and time of sports training also have a nonnegligible influence on the effect of sports training. Only regular, effective, and sufficient exercise training can excite patients with poststroke depression and reduce depression.

At present, exercise training is the main method for functional recovery of stroke. Its mechanism is to cause the correct functional reorganization of the brain through the characteristics of central nervous system plasticity changes and functional reorganization under job-guided exercise training [20, 21].

Sports training refers to exercises required for systemic or local aerobic metabolism and energy conversion for the purpose of enhancing physical fitness and improving brain function during various activities of the body. The effect of exercise training on rats is mainly reflected in improving disease resistance and adaptability and promoting the development of cerebellar cells.

Exercise training can significantly improve the cognitive ability of rats, and its main mechanism lies in the systematic and effective regulation of the body. After a training period, the regeneration of rat hippocampal neurons increased, the plasticity of the brain increased, and the HPA axis negative feedback regulation mechanism was redesigned. Physical exercise can significantly increase the activity of synaptophysin, promote the regeneration of dendrites, increase the number of dendrites, promote the formation of new synaptic connections, and activate static synapses. After a period of formal and orderly rehabilitation training, the degree of depression of the patient has decreased [22, 23].

## 3. Experimental Test

### 3.1. Experimental Animals

The experimental animals are 60 SD rats, between 220 and 250 g, free of specific pathogens, and healthy adult males. Laboratory facility certificate number: SYXK 2020-0005, ambient temperature 20-24°C, relative humidity 40%-50%, light and dark alternately for 10 h/14 h, and noise < 45 dB. Before the experiment, all rats were bred adaptively in a laboratory environment for one week.

### 3.2. Preparation of Rat PSD Model

The MCAO model rats were raised as orphans and received unpredictable chronic stress stimulation for 30 days. Unpredictable chronic stress stimuli include fasting, dehydration, tilting the squirrel cage to 45°, and swimming in ice water at 4°C for 5 minutes; continuous lighting for 15 hours in a humid environment for 1 day; and fixing the tail for 1 minute.

### 3.3. Experimental Method

Rats were divided into control group, sham group, PSD group, and PSD+ET group by random number table method, with 15 rats in each group. After the PSD model was successfully made, the rats in the normal training group and the intensive training group were trained on the animal experimental treadmill. Before formal training, rats should be adaptive training once a day with a treadmill speed of 4 m/min and then start formal training. PSD+ET group: on the first day, the treadmill speed is 4 m/min, and the rest is 30 s every 5 min; on the second day, the treadmill speed is 6 m/min, and the training time is 18 min; on the third day until on the 28th day, the treadmill speed is 8 m/min, and the training time is 24 min. The sham operation group and PSD group did not receive any rehabilitation training.

## 4. Test Results

### 4.1. The Basic Situation of Poststroke Depression

According to data surveys, patients with poststroke depression occur in the four stages of adolescence, youth, middle age, and old age. The site of occurrence is also in frontal lobe lesions, thalamus, occipital lobe, temporal lobe, pontine, medulla oblongata, and so on.

As shown in Figure 1, we can see that the disease often occurs in the elderly, but there are also a few teenagers who experience poststroke depression. Most of the occurrence sites are in frontal lobe lesions, with a 72% probability of occurrence.

### 4.2. Comparison of the Results of 3 Groups of Rats Behavioral Experiments

SPSS20.0 version software was used to analyze and process the experimental data, and the differences between the groups were compared by one-way analysis of variance. *P* < 0.05 indicates that the differences are statistically significant. According to Table 1, we can see that the sugar water consumption of the sham operation group before training was 72%, and the consumption increased gradually after training. The open field training before training stayed in the central area for 145 s, and after 15 days of training, it reached 152 s, but as the number of training days increased, it dropped to 141 s.

As shown in Figure 2, we can find that the sham operation group has different data trends before training, 15 days training, and 30 days after training. In the FST experiment before training, the immobility time of the sham operation group was about one minute, and the time was shortened after 15 days of training, and the time was extended after 30 days.

According to Table 2, we can see that the sugar water consumption of the PSD group before training was 53%, and the consumption after training was gradually reduced. The open field training before training stayed in the central area for 254 s, and after 15 days of training, it reached 265 s, but as the number of training days increased, it dropped to 259 s.

As shown in Figure 3, we can find that the trend of various data changes in the PSD group before training, 15 days after training, and 30 days after training is different. In the FST experiment before training, the immobile time of the PSD group was 114 s, and the time was increased after 15 days of training, and the time was shortened after 30 days.

According to Table 3, we can see that the sugar and water consumption of the ordinary training group before training is 56%, and the consumption after training decreases and then increases. The open field training before training stayed in the central area for 253 s, and after 15 days of training, it dropped to 240 s, and as the number of training days increased, it dropped to 213 s.

As shown in Figure 4, we can find that the trend of various data changes in the PSD group before training, 15 days after training, and 30 days after training is different. In the FST experiment before training, the immobile time of the PSD group was 114 s, and the time was increased after 15 days of training, and the time was shortened after 30 days.

### 4.3. Comparison of the Results of the IL-2/IL-6 of Rats in Each Group

According to Figures 5 and 6, compared with sham group, the expression of IL-2 and IL-6 in intestinal tissue and brain tissue in PSD group increased, and their expression levels decreased after exercise training intervention.

### 4.4. Expression of Intestinal Flora

According to Figure 7, compared with PSD group, the expression of Lactobacillus and Bifidobacterium increased after exercise training.

## 5. Discussion

Depression and stroke are two important causes of the socioeconomic burden. The World Health Organization recently reported that depression has “as a major cause of disability worldwide,” and stroke is one of the three major causes of the burden of disease [24]. The pathogenesis of PSD is still unknown, and there are many endogenous biological mechanisms and reactive source mechanisms that have been studied. It is believed that the disorder of intestinal flora after stroke is closely related to the development of PSD, while aerobic exercise can increase the colonization of probiotics and improve the composition and function of intestinal flora.

More evidence shows that exercise training is one of the nondrug therapies for poststroke depression. As a nondrug intervention measure before or after cerebral ischemia, exercise training has a good antidepressant effect, and exercise can increase the level of brain-derived neurotrophic factor (BDNF) in hippocampus [25, 26]. Long-term studies have shown that exercise training is more effective than antidepressants in preventing the recurrence of depression [27]. A recent clinical study showed that rTMS combined with aerobic exercise seems to be safe, feasible, and tolerable for individuals with a history of stroke and mild depressive symptoms. All participants had good compliance and showed improvement in depressive symptoms and walking ability [28]. Our study found that exercise training can effectively improve the depressive behavior of rats, especially in SPT, oft, and FST experiments.

There is a large and functional complex microbial community in the human gut, which encodes about 150 times the number of genes as the human genome, which is regarded as the human “second brain” [29]. With the deepening of the impact of gut microbes on human health and disease, exploring the relationship between gut microbiota and CNS function has become a hot topic. The intestinal flora can conduct two-way information communication with the brain through various pathways, including the nerve, endocrine, and immunity of the brain-intestinal axis and intestinal flora and stroke and its secondary CNS injury, anxiety, depression, autism, and Alzheimer's disease. The occurrence and development of a series of neuropsychiatric disorders are closely related to [30], among which, the relationship between stroke and depression and intestinal microflora is the current research hotspot.

Stroke can activate intestinal myeloid cells to trigger receptor-l to increase intestinal permeability and flora displacement [31]. We found that exercise training can reduce the expression of inflammatory factors in intestinal tissue and brain tissue, especially IL-2 and IL-6, promote the transformation of microglia into M2, inhibit neuroinflammation, and improve the occurrence of depression. In addition, the expression of Lactobacillus and Bifidobacterium increased after exercise training, which was similar to the previous results [32–34].

## 6. Conclusion

Stroke itself is a large, unpredictable stressful event that can lead to negative emotions in the patient. Stroke-induced dysfunction, family, and social status changes can also lead to patient mood changes, subsequently leading to the occurrence of PSD. Disorder of the gut microbiota also aggravates PSD production. PSD further aggravates the negative mood of patients and reduces their exercise enthusiasm. Experiments show that exercise training is a potential and effective method to improve PSD. Its mechanism may be related to inhibiting the expression of inflammatory factors and adjusting intestinal flora.

## Figures and Tables

**Figure 1:** Poststroke depression in different parts of different ages.

**Figure 2:** Behavioral experimental results of sham group.

**Figure 3:** PSD group behavioral experiment results.

**Figure 4:** Behavioral experiment results of PSD+ET group.

**Figure 5:** Protein expression results of intestinal tissue.

**Figure 6:** Protein expression results of brain tissue.

**Figure 7:** Expression of intestinal flora.

**Table 1:** Behavioral experimental results of sham group.

Mock surgical group	Count	SPT (%)	OFT (s)	FST (s)
Before training	8	72	145	63
Training for 15 days	4	74	152	61
Training for 30 days	4	75	141	65

Note: SPT refers to the sugar water consumption experiment, OFT refers to the open field experiment, and FST refers to the forced swimming experiment.

**Table 2:** PSD group behavioral experiment results.

PSD group	Count	SPT (%)	OFT (s)	FST (s)
Before training	8	53	254	114
Training for 15 days	4	52	265	116
Training for 30 days	4	51	259	110

**Table 3:** Behavioral experiment results of PSD+ET group.

Ordinary training group	Count	SPT (%)	OFT	FST
Before training	8	56	253	106
Training for 15 days	4	54	240	97
Training for 30 days	4	65	213	86

## Data Availability

The data underlying the results presented in the study are available within the manuscript.
